The article "Bone mesenchymal stem cells (BMSCs)-derived exosomal microRNA-21-5p regulates Kruppel-like factor 3 (KLF3) to promote osteoblast proliferation in vitro" was retracted in 2026. Reasons: original data or images not available; concerns about the data; concerns about the results or conclusions.

# Bone mesenchymal stem cells (BMSCs)-derived exosomal microRNA-21-5p regulates Kruppel-like factor 3 (KLF3) to promote osteoblast proliferation *in vitro*

**DOI:** 10.1080/21655979.2022.2067286

**Published:** 2022-05-13

**Authors:** Murong You, Zisheng Ai, Jihuan Zeng, Yang Fu, Liang Zhang, Xin Wu

**Affiliations:** a Department of Orthopedics, JiangXi Provincial People’s Hospital, Nanchang, Jiangxi Province, People’s Republic of China; b Department of Medical Statistics, Tongji University School of Medicine, Shanghai, People’s Republic of China

**Keywords:** Bone mesenchymal stem cells (BMSCs), exosomes, Kruppel-like factor 3 (KLF3), miR-21-5p, osteoporosis

## Abstract

Bone mesenchymal stem cells (BMSCs)-derived exosomes (Exos) play important roles in osteoporosis, while the regulation of microRNA (miR)-21-5p remains unclear. The BMSCs-derived exosomes were isolated from femoral bone marrow of trauma patients, which were then used to stimulate human osteoblasts (hFOB1.19 cells). The miR-21-5p mimic or inhibitor was transfected into BMSCs to overexpress or knockdown miR-21-5p. The functions of miR-21-5p in osteoporosis were assessed by cell counting kit-8 (CCK-8) assay, alkaline phosphatase (ALP) staining and alizarin red staining assays. We found that BMSCs-derived exosomes could enhance proliferation, osteoblastic differentiation and ALP activity of hFOB1.19 cells. BMSCs-derived exosomes with upregulated miR-21-5p could further enhance these protective impacts compared with that in BMSCs-derived exosomes, while BMSCs-derived exosomes with downregulated miR-21-5p reduced these cell phenotypes. MiR-21-5p could directly bind to the 3’-untranslated region (UTR) of Kruppel-like factor 3 (KLF3), and knockdown of KLF3 obviously attenuated these inhibitory effects of BMSCs-derived exosomes with downregulated miR-21-5p on osteoblastic differentiation and ALP activity of hFOB1.19 cells. In summary, BMSCs-derived exosomal miR-21-5p improved osteoporosis through regulating KLF3, providing a potential therapeutic strategy for osteoporosis.

## Highlight

- BMSCs-derived exosomes enhanced hFOB1.19 cell activities.
- MiR-21-5p participated in the protective role of exosomes in hFOB1.19 cells.
- MiR-21-5p regulated hFOB1.19 cell activities through targeting KLF3.

## Introduction

Osteoporosis is becoming a major public health issue along with the aging of the world’s population [1]. In China mainland, the population of osteoporosis still has a lower prevalence (approximately 13%) in comparison to that of other Caucasians [2]. Although potential therapeutic targets including non-coding RNAs (ncRNAs) and microRNAs (miRNAs) have been studied and identified [3], the development of promising therapeutic strategies are still necessary for the treatment of osteoporosis patients.

The article "Bone mesenchymal stem cells (BMSCs)-derived exosomal microRNA-21-5p regulates Kruppel-like factor 3 (KLF3) to promote osteoblast proliferation in vitro" was retracted in 2026. Reasons: original data or images not available; concerns about the data; concerns about the results or conclusions.

In recent years, the use of bone mesenchymal stem cells (BMSCs) is a promising cell treatment therapy for various human diseases including osteoporosis [4]. Exosomes (Exos) are secreted from BMSCs, which contain a reparative cargo carrying various miRNAs [5]. Increasing evidence has shown that these exosomes have the intercellular communication via delivering miRNAs to recipient cells [6,7]. Recent studies have focused on the protective roles of BMSCs-secreted exosomes on osteoporosis via inhibiting the expression of miRNAs-regulated mRNAs. For example, one study found that BMSCs-derived exosomes containing miR-424-5p attenuated osteogenic development [8]. Exosomal miR-186 derived from BMSCs was reported to enhance osteogenesis and then improve osteoporosis through regulating the hippo signaling in the postmenopausal osteoporosis model [9]. BMSCs-derived exosomes can enhance osteoblast proliferation through regulating miR-935 in the osteoporotic mouse model [10]. Interestingly, one recent study revealed that extracellular vesicles derived from adipose tissue stem cells could improve osteoporosis via miR-21-5p [11]. In addition, BMSCs-derived exosomes could enhance wound healing through the regulation of miR-21-5p [12]. Based on these findings, we hypothesized that BMSCs-derived exosomal miR-21-5p might also play a potential protective role in osteoporosis.

Kruppel-like factor 3 (KLF3), a member of the KLF transcription factor family, has been reported to modulate diverse physiological processes in different types of human tissue including angiogenesis, B lymphopoiesis, adipogenesis, erythropoiesis, myogenesis, and cardiac development [13–17]. Recently, it was found that inhibition of KLF3 might improve bone mass during osteogenesis [18], suggesting the possible involvement of KLF3 in osteoporosis. Interestingly, a recent study revealed that KLF3 was a target of miR-21-5p and participated in the regulation of miR-21-5p on the differentiation and activity of pancreatic cancer stem cells [19]. However, the regulatory mechanism of miR-21-5p and KLF3 in osteoporosis remains unclear.

In this study, we hypothesized that BMSCs-derived exosomes containing miR-21-5p might play a potential protective role in osteoporosis. The aim of this study was to investigate its role and the underlying regulatory mechanism.

## Materials and methods

### Isolation of bone mesenchymal stem cells (BMSCs)

Femoral bone marrow was donated from trauma patients. All patients signed the informed consent. BMSCs were isolated as previously described [20], and grown in (DMEM)/F-12 medium containing 10% fatal bovine serum (FBS) in a 37°C incubator with 5% CO_2_. The third-generation bone marrow mesenchymal stem cells that reached 80%-90% confluence were counted after trypsinization, and seeded on gelatin-coated 6 cells at a density of 5 × 10^3^ cells/cm^2^. Add 2 mL of α-MEM complete medium to the well culture plate, and place it at 37°C in vivo. The points were cultured in a 5% CO_2_ incubator, and after 24 h of cell adherent culture, aspirate the complete medium in the 6-well culture plate, and then add osteogenic, soft bone and adipogenic differentiation medium containing 10% fetal bovine serum α-MEM medium was used as a negative control at 37°C with a volume fraction of 5% CO_2_, cultured in an incubator, the medium was changed every 1 d. 2 weeks after adipogenic induction, the old medium in the culture plate was fixed with 40 g/L paraformaldehyde for 30 min, then aspirated and discarded. After 3 weeks of osteogenesis and chondrogenesis induction, the old medium in the culture plate was aspirated, fixed with 40 g/L paraformaldehyde for 30 min, and then aspirated and discarded. Alizarin red staining and toluidine blue staining were used to evaluate the osteogenesis, chondrogenic differentiation. Meanwhile, the morphology of BMSCs was observed by an inverted microscope after 3 d of culture. The BMSCs-related surface markers CD34 and CD90 were detected by flow cytometry using FITC-conjugated anti-CD31 (ab19361, abcam) and FITC-conjugated anti-CD90 (ab124527, abcam) as previously reported [21].

The article "Bone mesenchymal stem cells (BMSCs)-derived exosomal microRNA-21-5p regulates Kruppel-like factor 3 (KLF3) to promote osteoblast proliferation in vitro" was retracted in 2026. Reasons: original data or images not available; concerns about the data; concerns about the results or conclusions.

### Characterization of BMSCs-derived exosomes (Exos)

Exosomes were collected as previously described [22]. The exosomes-containing pellets were washed and re-suspended with PBS. The exosome concentrations were determined using the commercial bicinchoninic acid (BCA) kit. The exosomes morphology was observed by transmission electron microscopy (TEM), and exosomes-related surface markers CD9, CD63, and CD81 were analyzed by Western blot analysis.

### Cell transfection and treatment

Human osteoblasts (hFOB1.19 cells) were purchased from American Type Culture Collection (ATCC, Manassas, VA, USA). In addition, lentivirus-mediated short hairpin RNA (shRNA) targeting KLF3 (shKLF3), miR-21-5p mimics/inhibitor, and mimics NC/inhibitor NC were synthesized by Guangzhou Ribobio. For transfection, hFOB1.19 cells were seeded into a 12-well plate with (DMEM)/F-12 medium 24 h prior to treatment. When cell confluence reached approximately 70%, cells were resuspended with serum-free medium and seeded into the 12-well plates. Next, 500 ng of shKLF3, 100 nM of miR-21-5p mimics/mimics NC, miR-21-5p inhibitor/inhibitor NC were transfected into hFOB1.19 cells using Lipofectamine 2000 (Invitrogen) following the manufacturer’s instructions. After transfection, cells were grown at 37°C with 5% CO_2_. To evaluate the role of BMSCs-exosomes, 2 µg of exosomes was added into hFOB1.19 cells with approximately 1 × 10^5^ cells in six-well plates, followed by incubation for 12 h. Then, cell viability, alkaline phosphatase (ALP) activity, and osteoblastic differentiation were assessed.

The article "Bone mesenchymal stem cells (BMSCs)-derived exosomal microRNA-21-5p regulates Kruppel-like factor 3 (KLF3) to promote osteoblast proliferation in vitro" was retracted in 2026. Reasons: original data or images not available; concerns about the data; concerns about the results or conclusions.

### Cell counting kit-8 (CCK-8) assay

CCK-8 assay was performed as previously described [23]. In brief, approximately 1 × 10^5^ hFOB1.19 cells were plated into 96-well plates and cultured overnight. After treated with 2 µg of exosomes for 12 h, 10 ul CCK-8 reagent (Dojindo, Kumamoto, Japan) was added at different time points and incubated for another 2 h. Finally, a microplate reader was used to measure the absorbance at 450 nm.

### Alkaline phosphatase (ALP) and alizarin red staining

ALP staining and alizarin red staining assays were conducted as previously described [24]. For ALP staining, hFOB1.19 cells were cultured in fresh osteogenic differentiation medium containing 50 M ascorbic acid-2-phosphate, 10 mM β-glycerophosphate and 100 nM dexamethasone for 2 weeks. ALP staining was carried out using the commercial kit (Beyotime Institute of Biotechnology, Shanghai, China) following the manufacturer’s instructions. The ALP positive cells were analyzed using a microscope. For alizarin red staining, hFOB1.19 cells were stained by 2% alizarin red (pH = 4.2) for 15 min. After washing with distilled water twice, the mineralized nodules were examined with a phase contrast microscopy on the 21^st^ day.

### Cell cycle analysis

hFOB1.19 cells were seeded into 6-well plates and cultured for 24 h. Then cells were collected and washed with PBS twice. Cells were immobilized with precooled 70% ethanol, and RNase was added and incubated for 15 min. Then 50 μg/mL of propidium iodide (PI) (Bio-Rad, Hercules, CA, USA) was added to each well and incubated for another 30 min. Finally, cell cycle was detected by flow cytometry (BD Biosciences, Franklin Lakes, NJ, USA) as previously described [25].

### Luciferase reporter assay

The wild type (WT) or mutant (MUT) 3’-untranslated region (UTR) of KLF3 was cloned into psiCheck2 luciferase reporter vector. The hFOB1.19 cells were co-transfected with miR-21-5p mimics or mimics NC and recombinant luciferase vectors using Lipofectamine 2000 (Invitrogen) following the manufacture’s instruction. The relative luciferase activity was measured 2 days later using the dual luciferase reporter system as previously described [26].

### Quantitative reverse transcription-polymerase chain reaction (qRT-PCR)

Total RNAs were extracted by TRIzol reagent (TAKARA, Biotechnology, Dalian, Liaoning, China). The RNA concentration was determined by NanoDrop 2000 (Thermo Scientific, Waltham, Massachusetts, USA). The complementary DNA (cDNA) was synthesized using the PrimeScript RT reagent Kit (TAKARA Biotechnology, Dalian, Liaoning, China). The PCR reactions were performed using the Brilliant III Ultra-Fast SYBR Green qPCR Master Mix on an Agilent PCR-System. The relative expression levels of target genes were calculated using 2^−ΔΔCT^ method [27] with U6 snRNA and Glyceraldehyde-3-phosphate dehydrogenase (GAPDH) as the internal references. The primers were shown in Table 1.

The article "Bone mesenchymal stem cells (BMSCs)-derived exosomal microRNA-21-5p regulates Kruppel-like factor 3 (KLF3) to promote osteoblast proliferation in vitro" was retracted in 2026. Reasons: original data or images not available; concerns about the data; concerns about the results or conclusions.

**Table 1.** Primers

U6	F 5ʹ-CGCTTCGGCAGCACATATACTAAAATTGGAAC-3ʹ
	R 5ʹ-GCTTCACGAATTTGCGTGTCATCCTTGC-3ʹ
GAPDH	F 5ʹ-GGAGCGAGATCCCTCCAAAAT-3ʹ
	R 5ʹ-GGCTGTTGTCATACTTCTCATGG-3ʹ
miR-21-5p	F 5ʹ-GCCACCACACCAGCTAATTT-3ʹ
	R 5ʹ-CTGAAGTCGCCATGCAGATA-3ʹ
KLF3	F 5ʹ-TGTCTCAGTGTCATACCCATCT-3ʹ
	R 5ʹ-CCTTCTGGGGTCTGAAAGAACTT-3ʹ

F: Forward primer R: reverse primer

### Western blot analysis

Total proteins of cells were extracted using the RIPA Lysis Buffer following the manufacturer’s instructions. Approximately 50 μg protein samples were separated by 12% sodium dodecyl sulfate-polyacrylamide gel electrophoresis (SDS-PAGE), and then transferred to polyvinyl difluoride (PVDF) membranes. After blocking with 3% Bovine Serum Albumin (BSA), the membranes were incubated with primary antibodies CD63 (ab134045, abcam, 1:1,000), CD9 (ab92726, abcam, 1:2,000), CD81 (ab152267, abcam, 1:1,000), KLF3 (ab154521, abcam, 1:1,000), and GAPDH (ab8227, abcam, 1:1,000) at 4°C overnight. Then horseradish peroxidase (HRP) labeled goat anti-rabbit antibody to IgG (ab6721, abcam, 1:2,000) was added and incubated for 1 h. The protein complex was observed by an ECL kit (GE Healthcare Life Sciences) and analyzed using a Bio-Rad imaging system.

### Statistical analysis

Data were presented as the mean ± standard deviation (SD) using SPSS 21.0 software (IBM SPSS Inc. Chicago, IL, USA). The difference was explored by unpaired t test and one-way analysis of variance (ANOVA). P < 0.05 was considered as significant difference.

## Results

### Characterization of extracted BMSCs and exosomes (Exos)

To obtain the exosomes, BMSCs were isolated from femoral bone marrow of trauma patients and characterized. The extracted BMSCs showed a relatively homogeneous and vortex arrangement in the medium after 3 days of cultivation, and tended to be spindle shaped with clear boundaries and good refraction (Figure 1(a)). The purity of BMSCs was detected by flow cytometry. And 1.62% of CD34 (negative antigen) and 98.34% of CD90 (positive antigen) were detected, indicating a high purity of the isolated BMSCs (Figure 1(b)). Then the exosomes extracted from BMSCs were observed by electron microscope, and the diameter of these exosomes was about 40 nm (Figure 1(c)). To identify the exosomes, Western blot analysis was performed to detect the protein expression levels of exosome surface markers including CD9, CD63, and CD81 (Figure 1(d)), indicating that exosomes extracted from BMSCs could be used for the subsequent experiments.

The article "Bone mesenchymal stem cells (BMSCs)-derived exosomal microRNA-21-5p regulates Kruppel-like factor 3 (KLF3) to promote osteoblast proliferation in vitro" was retracted in 2026. Reasons: original data or images not available; concerns about the data; concerns about the results or conclusions.

**Figure 1.** The identification of BMSCs-derived exosomes. (a) The morphology of BMSCs by an inverted microscope. (b) Flow cytometry analysis of the BMSCs surface markers. (c) Exosomes were isolated from BMSCs under transmission electron microscopy (TEM) identification. (d) Western blot analysis of the exosome surface markers.

### BMSC-derived exosomes (BMSCs-Exos) enhanced the activity of hFOB1.19 cells

To evaluate the effects of BMSCs-exosomes (Exos) on hFOB1.19 cells, BMSCs-exosomes and hFOB1.19 cells were co-cultured, and then the relevant cell phenotypes were detected. After hFOB1.19 cells were co-treated by BMSC-Exos, cell viability of hFOB1.19 cells was detected at 24 h, 36 h, 48 h and 72 h, 96 h respectively. Our findings suggested that the cell viabilities of hFOB1.19 cells were remarkably elevated after BMSC-Exos treatment (Figure 2(a)). BMSCs-Exos significantly enhanced osteoblastic differentiation and alkaline phosphatase (ALP) activity of hFOB1.19 cells (Figure 2(b,c)). Subsequently, flow cytometry was performed to detect cell cycle and the results showed that BMSC-Exos treatment notably promoted cell cycle of hFOB1.19 cells with significant increased cell ratio of G2/M (Figure 2(d)). These results suggested that BMSC-Exos could enhance the activity of hFOB1.19 cells *in vitro*.

**Figure 2.** BMSCs-derived exosomes (Exos) enhanced the activities of hFOB1.19 cells. (a) hFOB1.19 cell proliferation determined by Cell counting kit-8 (CCK-8) assay after treated with BMSCs-derived exosomes at different time point. (b) Osteoblastic differentiation in hFOB1.19 cells evaluated by Alizarin Red staining after treated with BMSCs-derived exosomes. (c) Alkaline phosphatase (ALP) staining of hFOB1.19 cells after treated with BMSCs-derived exosomes. (d) hFOB1.19 cells cycle detected by flow cytometry after treated with BMSCs-derived exosomes. * *p* < 0.05, ** *p* < 0.01, *** *p* < 0.001, and NS indicates no significant difference.

### BMSCs-derived exosomes (BMSCs-Exos) with upregulated miR-21-5p further enhanced the activities of hFOB1.19 cells

To further investigate the impacts of exosomal miR-21-5p on hFOB1.19 cells, miR-21-5p mimics or inhibitor was transfected into BMSCs, and exosomes were isolated to stimulate hFOB1.19 cells. Firstly, the expression of miR-21-5p in BMSCs-Exos was detected by qRT-PCR, and the results showed that miR-21-5p mimics increased the expression levels of miR-21-5p in exosomes, while miR-21-5p inhibitor reduced its expression levels compared with that in the corresponding negative control (Figure 3(a)). Then CCK-8 assay was conducted and it showed that BMSCs-Exos with upregulated miR-21-5p obviously increased the cell viability of hFOB1.19 cells compared with that of BMSCs-Exos miR-NC, while BMSCs-Exos with downregulated miR-21-5p reduced the cell viability of hFOB1.19 cells compared with that of BMSCs-Exos inhibitor NC (Figure 3(b)). In addition, we observed more ALP positive hFOB1.19 cells in Exo-miR-21-5p mimic-treated group and less positive hFOB1.19 cells in Exo-miR-21-5p inhibitor-treated group (Figure 3(c)). BMSCs-Exos with upregulated miR-21-5p obviously promoted osteoblastic differentiation compared with Exos-miR NC, while BMSCs-Exos with downregulated miR-21-5p inhibited osteoblastic differentiation compared with Exos-inhibitor NC (Figure 3(d)). These results indicated that miR-21-5p participated in the protective role of BMSC-Exos on hFOB1.19 cell activities.

The article "Bone mesenchymal stem cells (BMSCs)-derived exosomal microRNA-21-5p regulates Kruppel-like factor 3 (KLF3) to promote osteoblast proliferation in vitro" was retracted in 2026. Reasons: original data or images not available; concerns about the data; concerns about the results or conclusions.

**Figure 3.** BMSCs-derived exosomes (Exos) enhanced the activities of hFOB1.19 cells via exosomal miR-21-5p. (a) Relative level of miR-21-5p in BMSCs-derived exosomes after transfection. (b) hFOB1.19 cell proliferation determined by Cell counting kit-8 (CCK-8) assay after treated with BMSCs-derived exosomes with changed miR-21-5p. (c) Alkaline phosphatase (ALP) staining of hFOB1.19 cells after treated with BMSCs-derived exosomes with changed miR-21-5p. (d) Osteoblastic differentiation of hFOB1.19 cells evaluated by Alizarin Red staining after treated with BMSCs-derived exosomes with upregulated or downregulated miR-21-5p. ** *p* < 0.01, *** *p* < 0.001.

### KLF3 was targeted by miR-21-5p

To investigate the regulatory axis of miR-21-5p, the downstream genes of miR-21-5p were predicted and verified. To screen the downstream targets of miR-21-5p that participated in osteogenesis, miR-21-5p mimics was introduced into hFOB1.19 cells, and the transfection efficiency was determined by qRT-PCR (Figure 4(a)). Targetscan was used to search the target genes of miR-21-5p, and the prediction showed that KLF3 might be a downstream gene of miR-21-5p (Figure 4(b)). The luciferase activity of WT-KLF3 was suppressed by miR-21-5p mimics compared with that of miR-NC in hFOB1.19 cells, while the luciferase activity of MUT KLF3 was not affected even if miR-21-5p was highly expressed (Figure 4(c)). The expression levels of KLF3 mRNA and protein were both measured in hFOB1.19 cells in different groups. The expression levels of KLF3 were reduced in miR-21-5p mimic transfected hFOB1.19 cells at both mRNA and protein levels, and were increased in miR-21-5p inhibitor transfected hFOB1.19 cells compared with that in their negative controls (Figure 4(d,e)). These results indicated that KLF3 was a target of miR-21-5p.

The article "Bone mesenchymal stem cells (BMSCs)-derived exosomal microRNA-21-5p regulates Kruppel-like factor 3 (KLF3) to promote osteoblast proliferation in vitro" was retracted in 2026. Reasons: original data or images not available; concerns about the data; concerns about the results or conclusions.

**Figure 4.** Kruppel-like factor 3 (KLF3) was targeted by miR-21-5p. (a) Relative level of miR-21-5p in hFOB1.19 cells after miR-21-5p mimics transfection. (b) The putative interaction predicted by Targetscan. (c) The impacts of miR-21-5p mimics on WT/MUT KLF3 in hFOB1.19 cells by luciferase reporter assay. (d and e) Relative level of KLF3 in hFOB1.19 cells after transfection of miR mimics or inhibitor determined by qRT-PCR (d) and western blot (e). * *p* < 0.05, ** *p* < 0.01, *** *p* < 0.001.

### Knockdown of KLF3 reversed the impacts of BMSCs-Exos with downregulated miR-21-5p on hFOB1.19 cell activities

Finally, rescue experiments were carried out to confirm the regulatory relationship between miR-21-5p and KLF3 on hFOB1.19 cell activities by treating hFOB1.19 cells with BMSCs-Exo with knockdown of KLF3. Firstly, qRT-PCR revealed that BMSCs-Exo shKLF3 significantly reduced the expression levels of KLF3 in hFOB1.19 cells at both mRNA and protein levels (Figure 5(a,b)). Then rescue experiments were performed and the data showed that BMSCs-Exos carrying miR-21-5p inhibitor significantly reduced ALP activity and osteoblastic differentiation of hFOB1.19 cells compared with BMSCs-Exos carrying inhibitor NC, BMSCs-Exos with knockdown of KLF3 enhanced the two cell phenotypes of hFOB1.19 cells, while co-treatment of BMSCs-Exo carrying miR-21-5p inhibitor and shKLF3 obviously attenuated the inhibitory effects of BMSC-Exos carrying miR-21-5p inhibitor on hFOB1.19 cell activities (Figure 5(b,c)). These data suggested that KLF3 participated in the regulation of exosomal miR-21-5p on hFOB1.19 cell activities.

**Figure 5.** KLF3 mediated the impacts of miR-21-5p on the activities of hFOB1.19 cells. (a and b) Relative mRNA (a) and protein (b) expression level of KLF3 in hFOB1.19 cells after treating with BMSCs-Exo sh-KLF3. (c and d) Alkaline phosphatase (ALP) staining (c) and osteoblastic differentiation (d) of hFOB1.19 cells after co-treated with BMSCs-derived exosomes (Exos) carrying miR-21-5p inhibitor and sh-KLF3. * *p* < 0.05, ** *p* < 0.01, *** *p* < 0.001.

## Discussion

Owing to the promising therapeutic potentials of stem cells-derived exosomes, extensive attention has been drawn to focus on their functions [28]. Recently, the exosomes secreted from BMSCs have been identified to exhibit various ameliorative roles against diverse types of diseased cells in human [29,30]. To increase our understandings of BMSCs-derived exosomes-related therapies, exploring the underlying molecular mechanisms are necessary. In this study, our data showed that BMSCs-derived exosomes with upregulated miR-21-5p could efficiently enhance cell proliferation, osteoblastic differentiation and ALP activity of hFOB1.19 cells, suggesting that BMSCs-derived exosomes might be a promising strategy for osteoporosis. The next challenge is how to deliver the BMSCs-derived exosomes into human body without any side effect, and this strategy might extend the window for osteoporosis treatment.

The article "Bone mesenchymal stem cells (BMSCs)-derived exosomal microRNA-21-5p regulates Kruppel-like factor 3 (KLF3) to promote osteoblast proliferation in vitro" was retracted in 2026. Reasons: original data or images not available; concerns about the data; concerns about the results or conclusions.

Firstly, we found that BMSCs-derived exosomes exhibited protective effects against osteoporosis through promoting osteoblast proliferation. The gain- and loss-of-function of miR-21-5p experiments confirmed that exosomal miR-21-5p derived from BMSCs played important roles in the protective effects of BMSCs-exosomes on osteoporosis. Previous studies reported that exosomal miR-21-5p derived from different types of stem cells had diverse biological activities. Exosomes containing miR-21-5p derived from MSCs could regulate macrophage polarization to improve myocardial reperfusion injury repair [31]. Cancer-derived exosomal miR-21-5p could induce angiogenesis and vascular permeability via the inhibition of KRIT1 [32]. Previous studies reported that miR-21-5p could reduce osteoclastogenesis in a *in vivo* osteoporosis model [33], and miR-21-5p also participated in the ameliorative functions of adipose tissue-derived stem cells secreted extracellular vesicles on osteoporosis [11]. However, the activity of BMSCs-derived exosomes, as well as exosomal miR-21-5p on osteoporosis remain unclear. Here, we confirmed the protective role of BMSCs-derived exosomes containing miR-21-5p on osteoporosis, which could contribute to the development of novel drugs targeting miR-21-5p.

Increasing evidence indicated that miRNAs play essential regulatory roles through directly binding to the 3’-UTR of their downstream mRNAs, followed by inhibition of translation [34,35]. To further understand the potential mechanisms of miR-21-5p on osteoporosis, we predicted the downstream target genes of miR-21-5p and identified KLF3, a well-known negative regulator of osteoporosis, and knockdown of KLF3 was reported to increase bone formation [18]. The data confirmed that KLF3 was one of the targets of miR-21-5p, and participated in the regulation of miR-21-5p on the cell differentiation and activities of pancreatic cancer stem cells [19]. Moreover, knockdown of KLF3 partially attenuated the inhibitory effects of BMSCs-derived exosomes with downregulated miR-21-5p on osteoblastic differentiation and ALP activity of human osteoblasts hFOB1.19 cells. These data also revealed that the miR-21-5p/KLF3 axis participated in the protective function of BMSCs-derived exosomes on osteoporosis. Our study further revealed that KLF3 participated in osteoblast proliferation, as well as the regulation of miR-21-5p on osteoporosis progression. Other downstream genes of miR-21-5p have also been reported in human diseases, such as SFRP5 in non‑alcoholic steatohepatitis [36], SMAD7 in lung cancer [37], PDCD4 in breast cancer [38], and LIFR in gastric cancer [39]. Whether these potential targets participated in the regulation of miR-21-5p on osteoporosis remains unclear, and our next plan is to investigate whether these downstream genes mediated the function of BMSCs-derived exosomal miR-21-5p on osteoporosis. In addition, a minor limitation in this study is that we only used one cell line (hFOB1.19 cells), and another or more cell lines should be selected to verify the regulatory model of miR-21-5p and KLF3 in the future.

The article "Bone mesenchymal stem cells (BMSCs)-derived exosomal microRNA-21-5p regulates Kruppel-like factor 3 (KLF3) to promote osteoblast proliferation in vitro" was retracted in 2026. Reasons: original data or images not available; concerns about the data; concerns about the results or conclusions.

## Conclusion

In summary, our study revealed that BMSCs-derived exosomes could enhance osteoblast proliferation, and then improve osteoporosis via miR-21-5p mediated inhibition of KLF3 (Graphical abstract). Our results provided a promising therapeutic target for osteoporosis.

## Supplementary Material

Supplemental Material

## Data Availability

The data that support the findings of this study are available from the corresponding author by reasonable request.
